The article "Azole Compounds as Inhibitors of Candida albicans: QSAR Modelling" was published in 2021. Journal: Front Chem.

# Azole Compounds as Inhibitors of *Candida albicans*: QSAR Modelling

**DOI:** 10.3389/fchem.2021.774416

**Published:** 2021-11-29

**Authors:** Davood Gheidari, Morteza Mehrdad, Mahboubeh Ghahremani

**Affiliations:** ^1^ Department of Chemistry, Faculty of Science, University of Guilan, Rasht, Iran; ^2^ Department of Chemistry and Biochemistry, Texas Tech University, Lubbock, TX, United States

**Keywords:** *Candida albicans*, QSAR, biological activity, MLR, benzimidazoles

## Abstract

*Candida albicans* is a pathogenic opportunistic yeast found in the human gut flora. It may also live outside of the human body, causing diseases ranging from minor to deadly. *Candida albicans* begins as a budding yeast that can become hyphae in response to a variety of environmental or biological triggers. The hyphae form is responsible for the development of multidrug resistant biofilms, despite the fact that both forms have been associated to virulence Here, we have proposed a linear and SPA-linear quantitative structure activity relationship (QSAR) modeling and prediction of *Candida albicans* inhibitors. A data set that consisted of 60 derivatives of benzoxazoles, benzimidazoles, oxazolo (4, 5-b) pyridines have been used. In this study, that after applying the leverage analysis method to detect outliers’ molecules, the total number of these compounds reached 55. SPA-MLR model shows superiority over the multiple linear regressions (MLR) by accounting 90% of the *Q* ^*2*^ of anti-fungus derivatives ‘activity. This paper focuses on investigating the role of SPA-MLR in developing model. The accuracy of SPA-MLR model was illustrated using leave-one-out (LOO). The mean effect of descriptors and sensitivity analysis show that RDF090u is the most important parameter affecting the as behavior of the inhibitors of *Candida albicans*.

## Introduction

Despite significant advances in medicinal chemistry, infectious illnesses caused by fungi continue to be a major danger to public health. Patients with serious diseases, such as neoplasia, and those receiving long-term full parenteral nutrition, should be extra careful. Despite the discovery of several successful antifungal medications over the last 3 decades, there are still unknown molecules with the properties needed to treat systemic yeast infections. As a result, finding new and more effective antimicrobial (Gheidari et al., 2020) medicines is critical, and most of the research program’s efforts are focused on developing new compounds. Miconazole and clotrimazole (Brincker, 1976; Smith, 1976; Rippon, 1982) are imidazole compounds that have demonstrated good clinical efficacy in dermatophytoses and nonsystemic candidiasis. Unfortunately, systemic miconazole usage has been linked to reversible thrombocytosis and anemia, whereas clotrimazole use has been linked to severe gastrointestinal problems. 2-(4-thiazolyl) benzimidazole (I) (thiabendazole)is another imidazole derivative with high clinical effectiveness in the treatment of dermatophytic infections in tropical areas. Since thiabendazole was shown to be useful in the treatment of a number of helmintic illnesses, a number of benzimidazole compounds have been tested for anti-infective properties. kThe most thoroughly investigated of these chemicals is 2-(a-hydroxybenzyl) benzimidazole (II) (HBB), which is a specific inhibitor of RNA-containing Enteroviruses.

The article "Azole Compounds as Inhibitors of Candida albicans: QSAR Modelling" was published in 2021. Journal: Front Chem.

HBB has no effect on viral adsorption, penetration, or un-coating, according to mechanism of action studies. Although the specific mechanism of this suppression is yet unknown, the major site of action of this antiviral drug appears to be inhibition of viral RNA synthesis. On the other hand, these drugs’ antiviral efficacy *in vivo* has been accompanied with symptoms of toxicity. One approach for modifying harmful effects and achieving the required selective activity is to apply structural changes to the basic molecule and create new derivatives or analogues. As a result, a novel series of benzoxazole and oxazolo(4,5-b) pyridine derivatives that are analogues of benzimidazole were investigated for antifungal activity against *Candida albicans* in this work, and their structures were revealed using instrumental analytical methods. One of the most important methods for predicting the biological activity of unknown compounds based on their molecular structures is quantitative structure-activity relationships (QSAR) (Konovalov et al., 2008). In QSAR/QSPR studies three considerations are very important, the first is the descriptors to ensure that they carry enough information of molecular structure for the interpretation of the activity property, the second is the modeling method employed and most importantly, the validation of QSAR models (Tetko et al., 2008). The use of internal and external validation has recently become a source of heated discussion (Roy et al., 2007). Internal validation is supported by one set of QSAR workers, whereas the other believes that internal validation is insufficient for testing model robustness and that external validation is required. Hawkins et al., the most vocal proponents of internal validation, believe that cross-validation may test model fit and examine whether predictions would hold true with new data not utilized in the model fitting process. They claim that when the sample size is small, keeping a portion of it back for testing is inefficient, and that it is far preferable to employ “computationally more burdensome” leave-one-out cross-validation instead. (Hawkins, 2003; Hawkins et al., 2003). For feature selection in this study, we utilized SPA (successive projections algorithm), which is a forward selection method that starts with one variable and adds a new one at each iteration until *N* variables are achieved (Hawkins, 2003). SPA is a strategy for selecting minimal collinearity subsets of variables and improving the conditioning of multiple linear regression (MLR) models. This technique was first presented for wavelength selection in spectroscopic data sets, particularly in cases when there is a lot of spectrum overlap (Araújo et al., 2001). It has been shown that MLR models obtained using SPA are superior to PLS models (Partial Least Squares) in various applications such as UV-VIS (Araújo et al., 2001; DantasFilho et al., 2005; Di Nezio et al., 2007; Grünhut et al., 2008), ICP-OES (Kawakami HarropGalvão et al., 2001), FT-IR (Honorato et al., 2005), and NIR spectroscopy (Breitkreitz et al., 2003; Filho et al., 2004). SPA has also been used in a number of classification studies (Pontes et al., 2005; Gambarraneto et al., 2009). The objective of this technique is to pick variables with the least amount of duplicate information content in order to overcome collinearity problems. The following are the SPA stages for the provided initial variable *k(0)* and the number *N*:

Step 0 *x*_*g*_ = *g*th column of data matrix X_train_; g = 1, . . . , *n*_c_ (prior to the initial iteration (n = 1)).

The article "Azole Compounds as Inhibitors of Candida albicans: QSAR Modelling" was published in 2021. Journal: Front Chem.

Step 1 *S* = {*g* such that 1 = *g* = *n*_*c*_ and  g∈ {*k*(0), . . . , *k*(*n*-1)}}, or, *S* stands for the set of variables that have yet to be chosen.

Step 2 The projection of *x*_*g*_ on the subspace orthogonal to *x*_*k(n-1)*_ *:*

$$Px_{g}=x_{g}-\left(x_{g}^{T}X_{k\left(n-1\right)}\right)x_{k\left(n-1\right)}{\left(x_{k\left(n-1\right)}^{T}x_{k\left(n-1\right)}\right)}^{-1}$$ (1)

For all g∈S , where **P** is the projection operator.

Step 3 *k(n)* = arg (max $\left\|Px_{g}\right\|$ ,  g∈S ).

Step 4
$Px_{g}$ ,  g∈S .

Step 5 *n* = *n* +1, and if *n* < N go back to Step 1.

End: The resulting variables are {*k(n); n* = 0, . . . , *N*-1}.

Figure 1 depicts the aforementioned processes for the initial iteration of SPA. The approach was originally designed to create multivariate calibration models (Araújo et al., 2001), but it was later broadened to address classification difficulties (Pontes et al., 2005).

**FIGURE 1:** Example of SPA with *n*_*c*_ = 4 and k (0) = 3. Result of the first iteration: k (Gheidari et al., 2020) = 1.

## Materials and Methods

### Data Set

Three classes of compounds investigated in this study are 2,5,6-trisubstituted benzoxazole (III), benzimidazoles(IV) 2-substituted oxazolo (4, 5-b) pyridine (V) derivatives (Yalçin et al., 2000). Figure 2 and Table 1 depicted the chemical structures and logarithmic experimental activity of these compounds. The IC50 activity parameter is a measure of antifungal potency that relates to the molar concentration of each chemical necessary to lower *Candida albicans* concentration by 50% when compared to the concentration measured in an infected culture. The 3D structures of the investigated compounds were optimized by means of semi-empirical quantum-chemical techniques of AM1 applied in the HyperChem computer software before computing the molecular descriptors (Hyperchem, 1993).

The article "Azole Compounds as Inhibitors of Candida albicans: QSAR Modelling" was published in 2021. Journal: Front Chem.

**FIGURE 2:** Structures of the benzoxazole, benzimidazoles and pyridine derivatives.

**TABLE 1:** Chemical structure, experimental activity and predicted activities of the *Candida albicans* inhibitors.

NO	Compound name	X	Y	Z	R	R_1_	R_2_	pIC50 exp	pIC50 pre
1	2-phenylbenzo[d]oxazole	CH	O	—	H	H	H	−1.2511	−0.9429
2	2−(4−tert−butylphenyl)benzo[d]oxazole	CH	O	—	C(CH_3_)_3_	H	H	−0.7824	−0.7398
3	4−(benzo[d]oxazol−2−yl)benzenamine	CH	O	—	NH_2_	H	H	−1.1135	−1.2878
4	4−(benzo[d]oxazol−2−yl)−N−methylbenzenamine	CH	O	—	NHCH_3_	H	H	−0.9931	−0.7232
5	5−chloro−2−(4−ethylphenyl)benzo[d]oxazole	CH	O	—	C_2_H_5_	Cl	H	−0.7308	−0.2049
6	N−(4−(5−chlorobenzo[d]oxazol−2−yl)phenyl)acetamide	CH	O	—	NHCOCH_3_	Cl	H	−0.5330	−0.2210
7	4−(5−chlorobenzo[d]oxazol−2−yl)−N−methylbenzenamine	CH	O	—	NHCH_3_	Cl	H	−0.7027	outlier
8	5−chloro−2−(4−chlorophenyl)benzo[d]oxazole	CH	O	—	Cl	Cl	H	−0.6630	outlier
9	5−chloro−2−(4−nitrophenyl)benzo[d]oxazole	CH	O	—	NO_2_	Cl	H	−0.5926	outlier
10	5−nitro−2−phenylbenzo[d]oxazole	CH	O	—	H	NO_2_	H	0.4257	0.5189
11	5−nitro−2−p−phenylbenzo[d]oxazole	CH	O	—	CH_3_	NO_2_	H	0.5375	0.6246
12	2−(4−tert−butylphenyl)−5−nitrobenzo[d]oxazole	CH	O	—	C(CH_3_)_3_	NO_2_	H	0.8256	0.2413
13	4−(5−nitrobenzo[d]oxazol−2−yl)benzenamine	CH	O	—	NH_2_	NO_2_	H	0.5461	−0.0056
14	2−(4−chlorophenyl)−5−nitrobenzo[d]oxazole	CH	O	—	Cl	NO_2_	H	0.6837	0.7435
15	2−(4−bromophenyl)−5−nitrobenzo[d]oxazole	CH	O	—	Br	NO_2_	H	0.9589	1.1683
16	2−(4−ethylphenyl)benzo[d]oxazol−5−amine	CH	O	—	C_2_H_5_	NH_2_	H	−0.8770	−1.4654
17	2−(4−fluorophenyl)benzo[d]oxazol−5−amine	CH	O	—	F	NH_2_	H	−0.9587	−1.1124
18	5−methyl−2−p−tolylbenzo[d]oxazole	CH	O	—	CH_3_	CH_3_	H	−1.001	−0.9365
19	2−(4−ethylphenyl)−5−methylbenzo[d]oxazole	CH	O	—	C_2_H_5_	CH_3_	H	−0.8856	−1.2869
20	2−(4−methoxyphenyl)−5−methylbenzo[d]oxazole	CH	O	—	OCH_3_	CH_3_	H	−0.8727	−0.5214
21	4−(5−nitrobenzo[d]oxazol−2−yl)benzenamine	CH	O	—	F	CH_3_	H	−0.9673	−0.3499
22	N−(4−(5−methylbenzo[d]oxazol−2−yl)phenyl)acetamide	CH	O	—	NHCOCH_3_	CH_3_	H	−0.6706	−0.8745
23	N−methyl−4−(5−methylbenzo[d]oxazol−2−yl)benzenamine	CH	O	—	NHCH_3_	CH_3_	H	−0.8770	−0.6418
24	N,N−dimethyl−4−(5−methylbenzo[d]oxazol−2−yl)benzenamine	CH	O	—	N(CH3)_2_	CH_3_	H	−0.7695	−0.4968
25	2−p−tolyloxazolo[4,5−b]pyridine	N	O	—	CH_3_	H	H	0.1806	−0.0856
26	2−(4−ethylphenyl)oxazolo[4,5−b]pyridine	N	O	—	C_2_H_5_	H	H	0.3010	1.1657
27	2−(4−methoxyphenyl)oxazolo[4,5−b]pyridine	N	O	—	OCH_3_	H	H	0.3182	0.2267
28	2−(4−ethoxyphenyl)oxazolo[4,5−b]pyridin	N	O	—	OC_2_H_5_	H	H	0.4300	1.1248
29	4−(oxazolo[4,5−b]pyridin−2−yl)benzenamine	N	O	—	NH_2_	H	H	0.1892	0.4186
30	2−(4−nitrophenyl)oxazolo[4,5−b]pyridine	N	O	—	NO_2_	H	H	0.4386	0.0819
31	2−(4−chlorophenyl)−5−nitrobenzo[d]oxazole	CH	O	CH_2_	H	H	H	0.1720	−0.3748
32	2−(4−methoxybenzyl)benzo[d]oxazole	CH	O	CH_2_	OCH_3_	H	H	0.4257	0.3954
33	2−(4−chlorobenzyl)benzo[d]oxazole	CH	O	CH_2_	Cl	H	H	0.4601	0.1951
34	2−(4−nitrobenzyl)benzo[d]oxazole	CH	O	CH_2_	NO_2_	H	H	0.5375	−0.0171
35	2−benzyl−5−chlorobenzo[d]oxazole	CH	O	CH_2_	H	Cl	H	0.4601	0.1356
36	2−(4−methoxybenzyl)−5−chlorobenzo[d]oxazole	CH	O	CH_2_	OCH_3_	Cl	H	0.6751	0.8628
37	2−(4−bromobenzyl)−5−chlorobenzo[d]oxazole	CH	O	CH_2_	Br	Cl	H	0.9761	1.2167
38	2−(4−nitrobenzyl)−5−chlorobenzo[d]oxazole	CH	O	CH_2_	NO_2_	Cl	H	0.7740	0.6188
39	2−benzyl−5−nitrobenzo[d]oxazole	CH	O	CH_2_	H	NO_2_	H	1.8317	1.5786
40	2−(4−methoxybenzyl)−5−nitrobenzo[d]oxazole	CH	O	CH_2_	OCH_3_	NO_2_	H	2.0381	1.5331
41	2−(4−bromobenzyl)−5−nitrobenzo[d]oxazole	CH	O	CH_2_	Br	NO_2_	H	2.3305	2.1263
42	2−(4−chlorobenzyl)−5−nitrobenzo[d]oxazole	CH	O	CH_2_	Cl	NO_2_	H	2.0682	1.8156
43	2−(4−nitrobenzyl)−5−nitrobenzo[d]oxazole	CH	O	CH_2_	NO_2_	NO_2_	H	2.1370	1.8988
44	5−methyl−2−(phenoxymethyl)benzo[d]oxazole	CH	O	CH_2_O	H	CH_3_	H	−0.8727	−0.9144
45	6−nitro−2−(phenoxymethyl)benzo[d]oxazole	CH	O	CH_2_O	H	CH_3_	H	−1.9391	−0.2366
46	5−chloro−6−nitro−2−(phenoxymethyl)benzo[d]oxazole	CH	O	CH_2_O	H	CH_3_	H	−1.7112	−1.3976
47	2−((4−chlorophenoxy)methyl)−5−chloro−6−nitrobenzo[d]oxazole	CH	O	CH_2_O	Cl	Cl	NO_2_	−1.5134	−1.9055
48	5−nitro−2−((phenylthio)methyl)benzo[d]oxazole	CH	O	CH_2_S	H	NO_2_	H	0.7568	0.5983
49	5−methyl−2−((phenylthio)methyl)benzo[d]oxazole	CH	O	CH_2_S	H	CH_3_	H	−0.7480	−0.1654
50	2−(phenoxymethyl)oxazolo[4,5−b]pyridine	N	O	CH_2_O	H	H	H	0.3311	0.0363
51	2−((p−tolyloxy)methyl)oxazolo[4,5−b]pyridine	N	O	CH_2_O	H	H	H	0.5848	0.3516
52	2−((4−chlorophenoxy)methyl)−5−methyl−1H−benzo[d]imidazole	CH	NH	CH_2_O	Cl	CH_3_	H	−0.6276	−1.2245
53	5−nitro−2−((phenylthio)methyl)−1H−benzo[d]imidazole	CH	NH	CH_2_S	H	NO_2_	H	0.7525	1.4148
54	5−methyl−2−((phenylthio)methyl)−1H−benzo[d]imidazole	CH	NH	CH_2_S	H	CH_3_	H	−0.7480	−0.9096
55	methyl 2−(phenoxymethyl)benzo[d]oxazole−5−carboxylate	CH	O	CH_2_O	H	COOCH_3_	H	−0.5545	−0.4934
56	methyl 2−((4−chlorophenoxy)methyl)benzo[d]oxazole−5−carboxylate	CH	O	CH_2_S	Cl	COOCH_3_	H	−0.3396	−0.6923
57	methyl 2−((4−chlorophenoxy)methyl)−1H−benzo[d]imidazole−5−carboxylate	CH	NH	CH_2_O	Cl	COOCH_3_	H	−0.3482	−0.2209
58	methyl 2−((phenylthio)methyl)−1H−benzo[d]imidazole−5−carboxylate	CH	NH	CH_2_S	H	COOCH_3_	H	−0.4600	−0.2282
59	5−nitro−2−phenethylbenzo[d]oxazole	CH	O	C_2_H_4_	H	NO_2_	H	0.6885	outlier
60	2−phenethyloxazolo[4,5−b]pyridine	N	O	C_2_H_4_	H	H	H	0.3671	outlier

The article "Azole Compounds as Inhibitors of Candida albicans: QSAR Modelling" was published in 2021. Journal: Front Chem.

### Molecular Descriptor

The most essential stage in any QSAR research is the identification and computation of structural descriptors as numerical encoded parameters defining chemical structures. The molecular descriptors in this study were created with Dragon program, version web 3.0 (Todeschini et al., 2003). Several QSAR studies have used the Dragon program to construct chemical descriptors. (Garkani-Nejad et al., 2004; González et al., 2004; González et al., 2005; Khalafi-Nezhad et al., 2005; Liu et al., 2006). Table 2 shows how the computed descriptors were split into 18 categories. It’s worth noting that calculating these descriptors is simple and quick. The average time to compute each structure was about 1 minute. This program has been used to produce a total of 1,497 descriptors for each molecule. For all molecules, descriptors with constant or very constant values were removed. Furthermore, pairs of variables with a correlation coefficient larger than 0.90 were identified as intercorrelated, and only one of them was used in the model development. After eliminating the descriptors with constant and intercorrelated values, a total of 327 descriptors were chosen for further research (Table 3).

**TABLE 2:** List of molecular descriptors that created by Dragon program.

Group name	Dimensionality	No. of descriptors	No. of descriptors in model
Constitutional descriptors	0	47	31
Functional groups	1	121	16
Atom−centered fragments	1	120	14
Empirical descriptors	1	3	2
Properties	1	3	2
Topological descriptors	2	266	42
Molecular walk counts	2	21	4
BCUT descriptors	2	64	7
Galvez topological charge indices	2	21	3
2D autocorrelation descriptors	2	96	18
Charge descriptors	3	14	9
Aromaticity indices	3	4	2
Randic molecular profiles	3	41	11
Geometrical descriptors	3	70	10
RDF descriptors	3	150	21
3D−MoRSE descriptors	3	160	23
WHIM descriptors	3	99	17
GETAWAY descriptors	3	197	25
Sum		1,497	257

**TABLE 3:** Selected descriptors of multiple linear regression.

Descriptor	Type of descriptor	Notation	Coefficient
Information Content index (neighborhood symmetry of 2−order)	Information	IC_2_	0**.**214
highest eigenvalue n. 8 of Burden matrix/weighted by atomic masses	BCUT	BEHm8	−0.295
quadrupole x−component value	Geometrical	Qxxe	0.27
Radial Distribution Function − 105	RDF	RDF105m	0.22
Radial Distribution Function − 050/weighted by van der Waals volume	RDF	RDF050v	0.285
signal 16/unweighted	3D−MoRSE	Mor16u	−0.673
signal 22/unweighted	3D−MoRSE	Mor22u	0.193
signal 32/unweighted	3D−MoRSE	Mor32u	0.41
signal 16/unweighted	3D−MoRSE	Mor16m	0.32
signal 13/unweighted	3D−MoRSE	Mor31m	0.416
2nd component accessibility directional WHIM index/weighted by van der Waals volume	WHIM	E2V	0.149
signal 30/weighted by van der Waals volume	3D−MoRSE	Mor30V	0.281

*R* ^*2*^_Cal_ = 0.96, *R* ^*2*^_Pre_ = 0.60, SE _Cal_ = 0.17, SE _Pre_ = 0.73, *F* = 6.675, REP % = 2.2.

The article "Azole Compounds as Inhibitors of Candida albicans: QSAR Modelling" was published in 2021. Journal: Front Chem.

### Regression Analysis

To choose a variable, a Stepwise-MLR technique is utilized. In biological systems, this technique has been utilized for variable selection and model building (Gupta et al., 2005; Leonard and Roy, 2006). The data set has been subdivided in two groups for regression analysis: training and prediction sets, and then a model is produced. In the present study, MLR model has been built by using 60 molecules. the results of statistical parameters: number of descriptors, correlation coefficient (R^2^), standard error (SE) and F statistic indicated that a series of molecules are very different from model, therefore, in the next stage, we identified outlier molecules. This is, in our view, the first QSAR research to identify outliers using a powerful and scientific method. The leverage analysis approach was utilized to detect outlier data. In order to identify outlier data, Leverage analysis method has been used (Despagne et al.,). In the first step, by making use of PCA, the *p*Cs which had the highest data variance were selected. Since the first two *p*Cs had the above-mentioned condition, they were selected as the main and most important PCs. After this step, Leverage graph was drawn based on the number of samples. As illustrated in Figure 3, samples of 7, 8, 9, 59, and 60 have more Leverage respectively compared to the rest of molecules and they were identified as outlier and omitted.

**FIGURE 3:** The Leverage graph based on the number of samples.

A trustworthy MLR model has strong R^2^ and F values, a low SE, and the fewest descriptors. Also, a high level of predictability should be present in the model. In addition, the model should have a high level of predictability. As a result, among the many models, the best model was picked, the characteristics of which are listed in Table 3. It is self-evident that as the number of descriptors grows, so does the R^2^. As illustrates in Figure 4, increasing the number of descriptors has an impact on R^2^ values.

The article "Azole Compounds as Inhibitors of Candida albicans: QSAR Modelling" was published in 2021. Journal: Front Chem.

**FIGURE 4:** The effect of the number of descriptors on the value of R^2^ in the Stepwise-MRL model.

From this figure one can see that the increase in the number of parameters up to twelve has a strong influence on the improvement of the correlation. As a consequence, we decided that twelve descriptors would be the best number of parameters to use. The descriptors IC_2_, BEHm8, Qxxe, RDF105m, RDF050v, Mor16u, Mor22u, Mor32u, Mor16m, Mor31m, E2V, and Mor30V exist in this model, and their meanings have been presented in Table 3. These descriptors’ formulas are not presented here for brevity’s sake; however, Dragon software can easily compute them (Todeschini and Consonni, 2000).

The correlation matrix (Table 4) shows that the selected descriptors have a significant degree of correlation, which is a problem for this model. In fact, Low-correlation descriptors should be utilized while creating a model, such that molecular descriptors reflect independent variables.

**TABLE 4:** Correlation matrix for the twelve chosen descriptors by means of Stepwise−MRL.

	IC2	BEHm8	QXXe	RDF105m	RDF050v	Mor16u	Mor22u	Mor32u	Mor16m	Mor31m	Mor30v	E2v
IC2	1	—	—	—	—	—	—	—	—	—	—	—
BEHm8	0.71289	1	—	—	—	—	—	—	—	—	—	—
QXXe	0.291867	0.449767	1	—	—	—	—	—	—	—	—	—
RDF105m	0.324553	0.366036	−0.21287	1	—	—	—	—	—	—	—	—
RDF050v	0.046017	0.325575	0.887022	−0.18233	1	—	—	—	—	—	—	—
Mor16u	−0.52103	−0.47151	−0.14793	−0.5522	0.151878	1	—	—	—	—	—	—
Mor22u	−0.04642	−0.10047	0.569542	−0.05905	0.558575	0.115754	1	—	—	—	—	—
Mor32u	0.339555	0.123565	0.448986	−0.50284	0.085389	−0.25631	0.324334	1	—	—	—	—
Mor16m	−0.26427	−0.3979	−0.51787	−0.17431	−0.35125	0.599117	−0.27855	−0.36023	1	—	—	—
Mor31m	−0.24366	−0.16379	0.339254	−0.49366	0.411267	0.179403	0.229171	0.227343	−0.35411	1	—	—
Mor30v	0.056618	−0.09594	−0.6632	0.325611	−0.47839	0.35268	−0.27186	−0.54116	0.522641	−0.52574	1	—
E2v	0.23577	0.498444	0.836901	−0.32191	0.658324	−0.18101	0.36587	0.600501	−0.58302	0.238531	−0.65492	1

## Results and Discussion

The major purpose of this study was to use SPA to select variables for MLR modeling by developing a QSAR model to estimate the activity parameter (pIC50) of compounds depicted in Figure 1 as *Candida albicans* inhibitors. It can be seen from this figure and Table 1 that the inhibitors of *Candida albicans* consisted of three different classes with very diverse substituents. As a result, the creation of a robust and interpretable QSAR model capable of properly predicting the pIC50 is required. As a first step, we created a linear MLR model, the parameters of which are listed in Table 3. This model was created with two objectives in mind. To begin, the appropriate variables were chosen using a Stepwise-MLR technique. Table 3 shows that out of 257 parameters, twelve descriptors of IC_2_, BEHm8, Qxxe, RDF105m, RDF050v, Mor16u, Mor22u, Mor32u, Mor16m, Mor31m, E2V, and Mor30V were chosen. These descriptors are classed as Information, BCUT, Geometrical, RDF, 3D-MoRSE, and WHIM descriptors. The Detailed descriptions of these descriptors are given in the literature (Todeschini and Consonni, 2000). The model’s second goal was to assess the linear connection between these characteristics and *Candida albicans* inhibitors’ biological activity. A value of 0.60 for *R* ^*2*^_Pre_ of this model reveals that it is able to account 60% of the variances of the pIC50. In reality, the Stepwise-MRL model is ineffective in predicting these compounds’ biological actions. Therefore, these results made us choose a more powerful method for selecting variables. In order to do this, successive projection algorithm was used final selection of descriptors. This study investigates the role of SPA-MLR, which has received little attention from scholars. In this method, at the first the descriptors which have the minimum correlation are selected and then, for final selection of the best model, the MLR method used. In the present study, by making use of this method, a model with thirteen descriptors as the final descriptors was selected whose statistical parameters and the name of its descriptors have been presented in Table 5.

The article "Azole Compounds as Inhibitors of Candida albicans: QSAR Modelling" was published in 2021. Journal: Front Chem.

**TABLE 5:** Statistical parameters and the name of descriptors in SPA−MLR model.

Descriptor	Type of descriptor	Notation	Coefficient
Moran autocorrelation of lag 8 weighted by van der Waals volume	2D autocorrelations	MATS8v	0.166586
Geary autocorrelation of lag 5 weighted by Sanderson electronegativity	2D autocorrelations	GATS5e	−0.23697
Geary autocorrelation of lag 7 weighted by Sanderson electronegativity	2D autocorrelations	GATS7e	−0.17958
Harmonic Oscillator Model of Aromaticity index	Geometrical	HOMA	−0.172
Radial Distribution Function − 090/unweighted	RDF	RDF090u	0.331935
Radial Distribution Function − 030/weighted by mass	RDF	RDF030m	−0.61428
signal 13/unweighted	3D−MoRSE	Mor13u	0.42232
signal 14/unweighted	3D−MoRSE	Mor14u	0.16831
signal 32/unweighted	3D−MoRSE	Mor32u	0.497132
signal 07/weighted by van der Waals volume	3D−MoRSE	Mor07v	−0.29036
signal 25/weighted by van der Waals volume	3D−MoRSE	Mor25v	−0.36172
leverage−weighted autocorrelation of lag 1/unweighted	GETAWAY	HATS1u	0.131395
H autocorrelation of lag 7/weighted by mass	GETAWAY	H7m	0.085106

SE_c_ = 0.30, R^2^ = 0.89.

There is no significant association between the selected descriptors, as seen in the correlation matrix (Table 6).

The article "Azole Compounds as Inhibitors of Candida albicans: QSAR Modelling" was published in 2021. Journal: Front Chem.

**TABLE 6:** The correlation matrix for the thirteen selected descriptors using SPA−MLR method.

	MATS8v	GATS5e	GATS7e	HOMA	RDF090u	RDF030m	Mor13u	Mor14u	Mor32u	Mor07v	Mor25v	HATS1u	H7m
MATS8v	1	—	—	—	—	—	—	—	—	—	—	—	—
GATS5e	−0.30741	1	—	—	—	—	—	—	—	—	—	—	—
GATS7e	−0.19173	−0.362	1	—	—	—	—	—	—	—	—	—	—
HOMA	0.230387	0.434716	0.019335	1	—	—	—	—	—	—	—	—	—
RDF090u	0.114087	−0.18651	0.010619	−0.73187	1	—	—	—	—	—	—	—	—
RDF030m	0.65665	−0.09176	0.366094	0.283897	0.21654	1	—	—	—	—	—	—	—
Mor13u	0.178512	−0.02735	0.518447	0.26828	−0.13945	0.606682	1	—	—	—	—	—	—
Mor14u	−0.04171	0.252716	−0.53748	−0.15829	−0.01353	−0.19766	−0.19999	1	—	—	—	—	—
Mor32u	0.003791	−0.03079	−0.44505	−0.30275	0.273409	−0.46963	−0.43707	0.091052	1	—	—	—	—
Mor07v	−0.03777	0.086135	0.019646	−0.3145	0.405478	0.105646	0.354031	0.31194	0.123109	1	—	—	—
Mor25v	−0.09809	0.477063	0.082629	0.173332	0.11963	0.349208	0.255182	0.201301	−0.07042	0.305127	1	—	—
HATS1u	−0.26587	−0.38164	−0.1431	−0.66778	0.094499	−0.51172	−0.08684	0.406374	0.202037	0.314072	−0.38987	1	—
H7m	0.419392	−0.25319	0.343601	0.35923	−0.03676	0.623623	0.286597	−0.11998	−0.13062	−0.23068	0.300966	−0.46849	1

The leave-one-out methodology was also utilized to demonstrate the stability of the model produced using the SPA-MLR method. The dataset (n = 55) was split into a training set of 41 compounds and a test (external assessment) set of 14 compounds using the process randomization approach. From the internal validation technique, the value of *Q*2 = 0.30 and RMSE = 0.74 was determined. The good results for the SPA-MLR model are not attributable to chance correlation or structural dependency of the training set, according to *Q*2 and RMSE values. Table 1 shows the observed and SPA-MLR predicted pIC50 values for all inhibitors of *Candida albicans* investigated in this study. The plot of the SPA-MLR predicted vs experimental pIC50 values for the data set is shown in Figure 5. A correlation coefficient of this plot indicates the reliability of the model.

**FIGURE 5:** Experimental pIC50 versus calculated pIC50 plot in internal validation.

The experimental values are plotted against the residuals of the SPA-MLR calculated values of pIC50 in Figure 6. The propagation of residuals on both sides of the line reveals zero error, indicating that the proposed model has no symmetric error.

**FIGURE 6:** Experimental pIC50 versus residual plot in internal validation.

In addition, the value of R^2^_pred_, REP and SEP was determined using the external validation approach, and these parameters were then utilized to determine the model predictivity. In this study, 25% of the data was chosen for external assessment. Table 7 displays the MLR result for comparing the SPA-MLR model. It can be seen from this Table that the statistical parameters of SEp, REP and *Q* ^*2*^_*LOO*_ have changed considerably. In fact, the SPA-MLR model beats the MLR model, making it ideal for predicting the pIC50 of *Candida albicans* inhibitors.

The article "Azole Compounds as Inhibitors of Candida albicans: QSAR Modelling" was published in 2021. Journal: Front Chem.

**TABLE 7:** Statistical results of SPA−MLR model compared to Stepwise−MRL model in external validation method.

	Q^2^	SE_P_	REP %
Stepwise−MRL	0.60	0.73	2.2
SPA−MLR	0.90	0.36	1.1

Figure 7 shows the residuals of the SPA-MLR computed pIC50 values in the external assessment technique displayed against the experimental values. The fact that the residuals propagate on both sides of the zero line suggests that the SPA-MLR model was developed without systematic error.

**FIGURE 7:** Experimental pIC50 versus residual plot in external validation.

Finally, we employed the suggested linear models to deduce the inhibitors of *Candida albicans’* mechanism of action. This implies we should look at the variables that are the most important predictors among the MLR model’s thirteen descriptors. Figure 8 shows the relative mean effect and sensitivity of each variable for the SPA-MLR models. The model show that RDF090u has a significant influence on biological activities of the *Candida albicans* inhibitors.

**FIGURE 8:** Relative mean effects for SPA-MLR model.

## Conclusion

The use of QSAR methods has been effective in establishing a mathematical link between inhibitors of *Candida albicans* and 2D autocorrelations, Geometrical, RDF, 3D-MoRSE, and GETAWAY. The results show that the SPA–MLR model outperforms the Stepwise-MRL models. This is because, unlike regression analysis, SPA–MLR allows for flexible mapping of the chosen characteristics by changing their functional dependency implicitly. This approach enabled us to develop a precise and relatively quick method for determining the IC50 of various antifungal derivative series, as well as to accurately estimate the IC50 of novel antifungal compounds.

## Data Availability

The original contributions presented in the study are included in the article/Supplementary Material, further inquiries can be directed to the corresponding authors.
